# Infantile colic, facts and fiction

**DOI:** 10.1186/1824-7288-38-34

**Published:** 2012-07-23

**Authors:** Abdelmoneim E M Kheir

**Affiliations:** 1 Department of Paediatrics, Faculty of Medicine, University of Khartoum, Khartoum, Sudan

**Keywords:** Colic, Crying, Infant, Baby

## Abstract

Infantile colic is one of the major challenges of parenthood. It is one of the common reasons parents seek medical advice during their child’s first 3 months of life. It is defined as paroxysms of crying lasting more than 3 hours a day, occurring more than 3 days in any week for 3 weeks in a healthy baby aged 2 weeks to 4 months. Colic is a poorly understood phenomenon affecting up to 30% of babies, underlying organic causes of excessive crying account for less than 5%. Laboratory tests and radiological examinations are unnecessary if the infant is gaining weight normally and has a normal physical examination. Treatment is limited and drug treatment has no role in management. Probiotics are now emerging as promising agents in the treatment of infantile colic. Alternative medicine (Herbal tea, fennel, glucose and massage therapy) have not proved to be consistently helpful and some might even be dangerous. In conclusion infantile colic is a common cause of maternal distress and family disturbance, the cornerstone of management remains reassurance of parents regarding the benign and self-limiting nature of the illness. There is a critical need for more evidence based treatment protocols.

## Introduction and definition

It is a behavioural syndrome characterized by excessive paroxysmal crying, that is most likely to occur in the evenings without any identifiable cause. There are so many definitions but the most widely used one is based on the amount of crying by Wessel et al. which states that it is paroxysms of excessive crying in an otherwise healthy baby lasting more than 3 hours per day, occurring > 3 days in any week for 3 weeks, aged 2 weeks to 4 months [1]. Rule of three.

Colic is one of the common reasons parents seek medical advice for their baby in his first 3–4 months of life. Those most affected by colic are the parents. Sleepless nights and the inability to console a newly arrived baby cause a great deal of stress, especially among first-time parents. Mothers of infants with colic were found to be more concerned about their infants’ temperament and even to feel rejection compared with mothers of infants without colic [2,3].

Colicky babies may be at an increased risk of abuse at the hands of exhausted and frustrated parents. Additionally, the parent may not properly bond with the child because of feelings of inadequacy and anger, leading to developing behavioral problems as the child grows [4].

The term colic derives from the Greek word kolikos or kolon, it is quite characteristic, a baby who has colic often cries about the same time every day, usually in the late afternoon or evening. Colic episodes may last from a few minutes to three hours or more on any given day. The crying usually begins suddenly and for no clear reason. The baby may have a bowel movement or pass gas near the end of the colic episode. Colic crying is intense and often high pitched. The face may flush, and he or she is extremely difficult — if not impossible — to comfort. Posture changes like Curled up legs, clenched fists and tensed abdominal muscles are common during colic episodes [5,6].

## Epidemiology

Internationally Colic affects 10-30% of infants worldwide. This condition is encountered in male and female neonates and infants with equal frequency. The colic syndrome is commonly observed in neonates and infants aged 2 weeks to 4 months. The incidence of colic in breastfed and bottle-fed infants is similar with no difference [7]. Increased susceptibility to recurrent abdominal pain, allergic disorders and certain psychological disorders may be seen in some babies with colic in their childhood. Illingworth found no association between the mother’s age, parity, or pregnancy history and colic [8].

## Aetiology

The cause of infantile colic remains unclear. Underlying organic causes of excessive crying must be considered during the evaluation. Organic causes account for less than 5 percent of infants presenting with excessive crying. These includes CNS causes like infantile migraine and subdural haematoma, GIT causes include constipation ,Cow’s milk protein intolerance, Gastro esophageal reflux ,Lactose intolerance, Intussusception, rectal fissure, strangulated inguinal hernia. Infections like Meningitis, Otitis media, Urinary tract infection and viral illness can also mimic colic. Trauma has to be excluded in a colicky baby namely child abuse, corneal abrasions, Foreign body in the eye, fractured bone and hair tourniquet syndrome [9,10].

Gastrointestinal, psychosocial, and neurodevelopmental disorders have been suggested as the cause of colic.

Gastrointestinal disorders have been implicated in colic because of the infant’s leg position and grimacing during a crying spell. Excessive crying or increased gas production from colon function can result in intraluminal gas formation and aerophagia. This mechanism does not appear to be the cause of colic, however, because radiographic images taken during a crying episode have shown a normal gastric outline [11]. Gut hormones such as motilin also may play a causative role in colic. Motilin is thought to cause hyperperistalsis, leading to abdominal pain and colic [12].

Although studies have addressed possible psychosocial causes of colic, no evidence has been found in support of this mechanism. Even when colicky infants are cared for by trained occupational therapists, they cry twice as long as infants without colic. The hypothesis that colic is an early manifestation of a difficult temperament is not supported by prospective longitudinal studies [13,14].

Studies have suggested that colic may lie at the upper end of the normal distribution of crying in infants. The fact that most infants outgrow colic by four months of age lends support to a neurodevelopmental cause of colic [9].

New epidemiologic evidence suggests that exposure to cigarette smoke and its metabolites may be linked to infantile colic. Moreover, studies of the gastrointestinal system provide corroborating evidence that smoking is linked to increased plasma and intestinal motilin levels and higher-than-average intestinal motilin levels are linked to elevated risks of infantile colic [15].

## Work up

Colic is a common condition in early infancy that causes a great deal of concern. Parents and caregivers should be encouraged to document crying and fussing spells for review by the physician. A period of wellness followed by specific periods of crying is reassuring. Diagnosis is by exclusion. Further workup should be considered in infants who have frequent regurgitation of more than 28 g (1 oz), apneic or cyanotic episodes, fever, respiratory difficulties, poor weight gain, or abnormal findings on neurologic examination. Serial examination of the infant during times of the day when the infant is less fussy may be necessary [16-18].

Laboratory tests and radiographic examinations usually are unnecessary if the child is gaining weight normally and has a normal physical examination [19].

If the patient’s stools are excessively watery, testing them for excess reducing substances (Clinitest) may be worthwhile. If results are positive, this may be an indication of an underlying GI problem, such as acquired (post infectious) lactose intolerance. Stool may be tested for occult blood to rule out cow’s milk allergy.

Mothers often believe that their baby’s crying may be related to milk formula or disease which can be managed by changing the infant’s formula from cow’s milk to a soya protein or casein hydrolysate formula. When a formula was changed, mothers more frequently believed that the cause of the problem was intrinsic to the child (P<0.001) and that their infant had had a “disease or illness” (P<0.001). When formula changes occurred, 26% of mothers believed that their infants were allergic to cow milk. These beliefs may affect a mother’s perceptions of her child’s vulnerability [20].

## Treatment

The mainstay of colic management is an acknowledgment by the physician of the difficulties the parents are facing and an inquiry into the well-being of the parents [21]. The single most effective step remains reassurance of parents regarding the benign and self-limiting nature of the illness as most of the babies improve by the age of 3 to 4 month. Drug treatment generally has no place in the management of colic, unless the history and investigations reveal gastro esophageal reflux.

Simethicone, a safe, over-the-counter drug for decreasing intraluminal gas, it is a non absorbable medication that changes the surface tension of gas bubbles, allowing them to coalesce and disperse and releasing the gas for easier expulsion. It has been promoted as an agent to decrease colicky episodes. A randomized, placebo-controlled, multicenter trial concluded that treatment with this agent produces results similar to those of placebo. The perceived improvement may be a placebo effect. Two other RCTs found no benefit for treatment with simethicone [22].

Dicyclomine hydrochloride is an anticholinergic drug that has been proven in clinical trials to be effective in the treatment of colic. However, because of serious, although rare, adverse effects (eg, apnea, breathing difficulty, seizures, syncope), its use cannot be recommended [23]. Cimetropium bromide, which is widely used in Italy to treat infantile colic, showed a decrease in duration of crying crises in the treated group compared with placebo. The major side effect was sleepiness; there were no reports of life-threatening events [24].

Dietary changes like eliminating cow’s milk proteins is indicated only in cases of suspected intolerance to the protein (eg, positive family history, eczema, onset after the first month of life, association with other GI symptoms such as vomiting or diarrhea). In infants with suspected allergy to cow’s milk protein (formula fed) a protein hydrolysate formula is indicated. Extensively hydrolyzed protein formulas may reduce colic, while partially hydrolyzed formulas should not be used in infants with colic due to cow’s milk protein allergy [25].

Use of soy-based formula is not recommended because many infants allergic to cow’s milk protein may also develop intolerance to soy protein. if the mother is breastfeeding, a period of elimination of allergenic foods (e.g. dairy, nuts, soy, citrus, etc.) from her diet in order to observe changes in the baby’s condition. If the crying is related to a cow’s milk allergy benefits are usually seen within 2–7 days [26-28].

Hill et al. suggested that a period of dietary modification with a low allergen diet and appropriate nutritional support should be considered in healthy infants with colic .He also found that exclusion of allergenic foods from the maternal diet was associated with a reduction in distressed behavior among breastfed infants with colic presenting in the first 6 weeks of life [29,30].

In some patients, exercise-induced anaphylactic reactions (EIAN) occur only when a particular food is eaten before exercise. Food-exercise combined challenge may be useful in identifying foods that favor exercise-induced anaphylactic reactions in children with multiple food-dependent EIAn [31,32].

Probiotics may have a role in treatment of infantile colic. Lactobacillus reuteri endogenous to the human GI tract was found to relieve colic symptoms in breastfed infants within one week of treatment. In a more recent study, 50 exclusively breastfed colicky infants were randomly assigned to receive either L reuteri or placebo daily for 21 days. A 50% reduction in crying time from baseline was noted in the L reuteri group compared with the placebo group on days 7. The study concluded that L reuteri at a dose of 108 colony-forming units per day improved symptoms of infantile colic and was well tolerated and safe. Further studies are needed before this can be recommended as a routine therapy for colic in infants [33,34]. Recently as revised by Critch there is insufficient evidence to recommend for or against the use of probiotics or prebiotics in the management of colic [35].

## Alternative medicine

Oral hypertonic glucose and sterile water were compared for treatment of colic in infants in a randomized trial. In the group receiving glucose, 30% had significantly less colic than the placebo group [36].

Herbal teas containing mixtures of chamomile, vervain, licorice, fennel, and lemon balm, used up to three times a day (150 mL per dose) have been shown to decrease crying in colicky infants. Given the multiplicity of herbal products, the lack of standardization of strength and dosage, and potential interference with normal feeding, parents should be cautioned about their use [37,38].

Spinal manipulation is a traditional form of treatment practiced by chiropractors, osteopaths, physiotherapists and other healthcare providers mostly (but not exclusively) to treat musculoskeletal problems. Spinal manipulation can be described as ‘the use of hands applied to the patient incorporating the use of instructions and maneuvers to achieve maximal painless movement and exposure of the musculoskeletal system. Evidence for the efficacy of spinal manipulation in treating infantile colic is inconclusive. Physicians should be cautious about recommending spinal manipulations in infants [39,40].

Rhythmic calming techniques are effective in calming colicky babies which forms the core of the 5 Ss approach.

1. Swaddling, safe swaddling carefully avoiding overheating, covering the head, using bulky or loose blankets, and allowing the hips to be flexed [41,42].

2. Side or stomach (holding a baby on the back is the only safe position for sleep, but it is the worst position for calming a fussy baby);

3. Shhh sound (making a strong shush sound near the baby's ear [43,44].

4. Swinging the baby with tiny jiggly movements (no more than 1" back and forth) always supporting the head and neck [44,45]

5. Sucking (Letting the baby suckle on the breast, your clean finger or a pacifier)

Numerous studies mentioned above have shown that when key components of the “5 S’s” (e.g. swaddling, shushing, swinging) are used all night they can improve sleep or reduce crying; and, when the “5 S’s” are done correctly and in combination, they offer significant potential to promptly reducing infant crying and promote sleep.

Remind parents about the importance of feeding a hungry baby, changing wet diapers, and comforting a baby who is cold and crying as a result of these factors. Soothing music accompanied with parental attention (including eye contact, talking, touching, rocking, walking, and playing) may be effective in some infants and is never harmful.

Encourage parents to discuss their feelings and concerns with each other to obtain support. Emphasize the responsibility of the whole family in the care of a baby with colic.

## Conclusion

Infantile colic is a common cause of maternal distress and family disturbance, the cause remains unclear, the cornerstone of management remains reassurance of parents regarding the benign and self-limiting nature of the illness as most of the babies grow out of it by the age of 3–4 months. Investigations are rarely required and drug treatment is usually ineffective. Consistent follow up and a sympathetic physician forms the basis of management in patients with colic. There is a critical need for more evidence based treatment protocols.

## Competing interests

The author declares that he has no competing interest.
